RETRACTED

# Study on the Correlation between the Prevalence of Venous Thromboembolism in Kazak Pregnant and Lying-In Women in Xinjiang

**DOI:** 10.1155/2022/7001743

**Published:** 2022-08-04

**Authors:** Guanglei Tian, Hongbo Ci, Wei Song, Bing Zhu, Xiong Chen, XiaoHu Ge

**Affiliations:** ^1^Graduate School, Xinjiang Medical University, Urumqi 830054, China; ^2^Department of Hepatobiliary Surgery, People's Hospital of Xinjiang Uygur Autonomous Region, Urumqi 830011, China; ^3^Department of Vascular Surgery, People's Hospital of Xinjiang Uygur Autonomous Region, Urumqi 830001, China

## Abstract

In order to reveal the correlation between the prevalence of venous thromboembolism in Kazak pregnant and lying-in women in Xinjiang, the polymorphisms in the promoter region and coding region of the TAFI gene and the interaction of environmental factors are investigated. In this study, determination and analysis of anticoagulation indexes are conducted. The activity of antithrombin III and protein C is measured by chromogenic substrate method, and the activity of protein S is measured by coagulation method. Besides, the detection of APC-R is performed by APC-APTT method. The experimental results show that the prevalence rate of hereditary thrombophilia + DVT among Kazak pregnant women in Xinjiang is 33.8%, and the prevalence rates of AT-III deficiency, PC deficiency, PS deficiency, APCR, and Hcy are 17.5%, 16.7%, 22.0%, 23.7%, and 26.8%, respectively. Also, the genotype frequency and allele frequency distribution of each group are in line with Hardy–Weinberg equilibrium (*P* > 0.05). The comparison result indicates that the gene frequency has reached a genetic balance and is representative of the population. It is clearly evident that the polymorphisms of prothrombin gene rs3136447 and rs5896 may be associated with hereditary thrombophilia in Xinjiang Kazaks.

## 1. Introduction

Venous thromboembolism (vte), including deep vein thrombosis (DVT) and pulmonary embolism (PE), are two clinical manifestations of the same disease at different sites and stages [1]. There are many systematic theories about thrombosis, and the most classical one is the “Virchow triangle.” It refers to the three elements of thrombosis: blood stasis, vascular wall injury (or endothelial injury), and hypercoagulable state [2, 3]. For arteriovenous fistulas, blood stasis is related to blood flow velocity or blood flow. Generally speaking, for autogenous arteriovenous fistulas, blood flow less than 300 ml/min and artificial vascular fistulas less than 600 ml/min may lead to blood stasis. However, it should be noted that the threshold is not an absolute value in the strict sense, and there are certain individual differences. The blood flow threshold of thrombosis is a very important indicator to determine the blood flow monitoring of internal fistula [4]. According to the existing clinical research and statistics, VTE is one of the main causes of maternal mortality, and its annual incidence is between 1‰ and 2‰ [5]. Three elements of Virchow thrombosis, blood stasis, endothelial injury, and hypercoagulable state, often occur in obstetrics and gynecology patients, so the incidence is higher than that of the general population. It has been reported in the literature that the incidence of venous thromboembolism in the obstetric population is 0.06% to 1.8%, while the incidence of DVT in gynecological surgery patients without preventive medication can reach 14% to 40% [6]. Previous studies have shown that the Kazak population in Xinjiang has genetic factors for venous thromboembolism. Preliminary studies have shown that the activities of protein C (PC) and protein S (PS) in Kazak pregnant and lying-in women are lower than those in Han women, which may be an important factor in their susceptibility to venous thrombosis before and after childbirth [7].

RETRACTED

There was no report of venous thromboembolism among Kazak pregnant women in Xinjiang. The incidence of venous thromboembolism in Kazak pregnant women in Xinjiang and the relationship between the causes of venous thromboembolism in Kazak women and environmental and genetic factors need to be further studied [8]. It is of great significance to explore the pathogenesis of venous thromboembolism in Kazak women in Xinjiang and improve the prevention and treatment of venous thromboembolism in Kazak pregnant women. In this study, the detection of antithrombin-III (AT-III), PC, PS, and activated protein C resistance (APCR) and gene identification methods are employed to identify the DNA of the selected genes [9]. Through the analysis of the relationship between anticoagulant protein deficiency, candidate genes, and Kazak pregnant women in Xinjiang, the possible interactions between genes and genes and environment can be further analyzed. These results can provide valuable guidance for clinical prevention and treatment of such diseases.

This paper is organized as follows: Section 2 discusses the related work, and Section 3 presents the experimental materials and methods. In Section 4, the experimental results and analysis are proposed. Finally, in Section 5, some concluding remarks are made.

## 2. Related Work

Venous thrombosis in pregnant women is mainly due to the presence of hypercoagulable state in pregnant women. And with the increase of fetus and abdominal pressure, some patients may not exercise often, which will cause slow blood flow [10, 11]. Hypercoagulable state and slow blood flow are risk factors for venous thrombosis. Studies have shown that VTE is a multifactorial disease caused by the interaction of genetics and environmental exposure. Many patients with VTE have one or more genetic predisposing factors, and epigenetic changes are also an important cause of VTE [12]. Genetic risk factors of VTE are highly heterogeneous, with significant differences in risk weight and independence. In terms of mechanism [13], VTE genetic defects can be roughly divided into four categories, including (1) loss of function (LOF) of coagulation inhibitor gene, such as variation of antithrombin gene, protein C gene, protein S gene, and thrombomodulin gene (THBD), which can lead to weakening of anticoagulant system function; (2) gain of function (GoF), such as partial variation of prothrombin gene (F2) G20210 A, factor V gene (FV) Leiden, von Willebrand factor (VWF), and factor VIII (F8), which can enhance the trend of blood coagulation; (3) abnormal gene function of fibrinolytic system, such as plasminogen activator inhibitor-1 gene (PAI-1) 4 g/5 g, which can lead to inhibition of fibrinolytic system function; (4) other gene variations or epigenetic changes that may indirectly affect blood coagulation, such as high DNA methylation levels, and may lead to the silencing of a variety of anticoagulant factors [14, 15].

RETRACTED

Statistical analysis of the polymorphisms in the promoter region and coding region of the TAFI gene showed that the polymorphisms of the prothrombin gene rs3136447 and rs5896 may be related to the hereditary thrombophilia of the Kazaks in Xinjiang [16]. The rs3136447 and rs5896 loci are located in the 4th intron and 6th exon of chromosome 11, respectively. In recent years, people have made remarkable progress in understanding the function of introns; in particular, the mechanism by which introns regulate gene expression has begun to be revealed [17]. Studies have suggested that introns are likely to be actively involved in regulating tissue-specific expression of genes. The mutation of rs3136447 and rs5896 may affect the transcription and production of prothrombin, thus directly participating in the process of coagulation and anticoagulation, but further confirmation by functional studies is needed [18]. In recent years, the interaction analysis between environmental factors and disease candidate gene polymorphisms has received more and more attention with the development of molecular epidemiology. There is no report on the interaction between prothrombin gene mutation and environmental factors in patients with hereditary thrombophilia [19]. Therefore, hereditary thrombophilia may be caused by the interaction of multiple genes and complex environmental factors. Some scholars have proposed that the mutation or defect of each gene may have only a weak effect on the susceptibility of disease or may not be enough to cause disease, so it is necessary to carry out site-site, gene-gene, and gene-environment interactions.

RETRACTED

From the perspective of the patient's environmental factors, the prevalence of Imchen stage genetic related venous thromboembolism deserves further analysis [20]. In some populations with different characteristics, there are significant differences in the prevalence of Imchen phase genetic related venous thromboembolism, such as the age and fresh vegetable intake. Among Kazak pregnant women, the prevalence of hereditary thrombophilia and/or VTE increased with age, and the prevalence is higher in the age group over 35 years of age [21]. At the same time, the intake of fresh vegetables decreased and the intake of fresh meat increased. In addition, there are no significant differences in the prevalence of hereditary thrombophilia among the groups in the history of hypertension, drinking water, fresh fruit intake, and salted meat intake [22]. And through the univariate analysis, it is found that the three factors of age, fresh meat intake, and fresh vegetable intake are all retained in the model, and the influence trend of age and fresh meat intake is consistent with the univariate analysis results. The clinical analysis may be related to the adjustment of maternal diet structure.

## 3. Experimental Materials and Methods

### 3.1. Experimental Materials

The sample populations are all pregnant and lying-in women of the right age among the resident Kazak population in Xinjiang Kazakh Autonomous Prefecture. A cross-sectional survey of pregnant women who are over 20 years old in Xinjiang Kazakh Autonomous Prefecture is performed. The pregnant and lying-in women should be excluded with following factors: age <20 years, severe liver disease, varicose veins, diabetes, heart failure, nephrotic syndrome, and polycythemia vera. The survey is conducted after the subjects signed the informed consent. Finally, 976 Kazak pregnant and lying-in women volunteers are obtained, with an average age (27.22 ± 8.4).

The instruments are as follows: centrifuge (Eppendorf), D-37520 desktop centrifuge (Thermo), PCR machine (GeneAmp PCR System 9700, Applied Biosystems), MassARRAY TM Nanodispenser (SAMSUNG), MassARRAY compact System (SEQUENOM), G384 + 10 Spectrochip™ (SEQUENOM), and pipette (Eppendorf).

The specific reagents include HotStarTaq DNA Polymerase (1000 U) (including 4 × 250 units HotStarTaq DNA Polymerase, 10 × PCR Buffer, 25 mM MgCl2, Qiagen Company), iPLEX TM Reagent Kit (including 10 × SAP Buffer, 1 U/*μ*L SAP enzyme, 10 × iPlex Buffer, iPlex Termination mix, iPlex enzyme, SEQUENOM Company), Clean Resin (SEQUENOM Company), and dNTP Mixture (TaKaRa Company).

RETRACTED

### 3.2. Proposed Methods

#### 3.2.1. Venous Blood Collection Method

Venous blood is collected during venous blood collection, anticoagulated with 0.109 mol/L sodium citrate 1 : 9, centrifugation radius 8 cm, centrifuged at 3000 r/min for 10 min, and the plasma is stored at −80°C and transported under frozen conditions. For determination of special indicators, genetic DNA is extracted from anticoagulated whole blood using standard methods.

#### 3.2.2. Determination of Blood Indexes

For AT-III, PS, PC, APC-R, and Hcy, thaw in a 37°C water bath before use, centrifuge at 2000 r/min for 20 minutes at room temperature to avoid cold activation of platelets, and separate plasma; must ensure that platelets are removed. The activities of antithrombin III and protein C are measured by the chromogenic substrate method, the activity of protein S is measured by the coagulation method, and the detection of APC-R is performed by the APC-APTT method.

#### 3.2.3. Questionnaire Survey

The general conditions of the research subjects (history of hypertension, drinking water, consumption of fresh meat, consumption of fresh vegetables, consumption of fresh fruits, consumption of salt, and salted meat) are asked.

#### 3.2.4. Statistical Methods

The correlation analysis between FII gene polymorphism and genetic inheritance of Kazak pregnant and lying-in women with venous thromboembolism in the pregnancy period is achieved by comparing the allele frequency and genotype frequency between the case group and the control group, and the *χ*^2^ test is used. The linkage disequilibrium of the three polymorphic loci is calculated by Haploview 4.3 software. The Hardy–Weinberg equilibrium test is performed on the three candidate loci of FII using plink software [23].

The correlation analysis between FV gene polymorphism and AT-III deficiency, PC deficiency, and protein S deficiency in Kazak population is conducted. Fisher's exact test assesses differences between groups of categorical variables. Differences in genotype frequencies between groups are assessed by the Mantel–Haenszel chi-square test and Fisher's exact test. Logistic regression models estimated odds ratios (ORs) and 95% confidence intervals (CIs). *P* < 0.05 is considered to be statistically significant. Hardy–Weinberg equilibrium test analysis is performed on the five candidate sites of FV using Plink software.

#### 3.2.5. Genotyping Method

In order to explore the polymorphisms in the promoter region and coding region of the TAFI gene, the candidate genes selected for gene screening and genotype identification in this study are FII gene, FV gene, FXI gene, F XII gene, F XIII gene, MTHFR gene, ABO Gene non-O type, SERPINC1 gene, SERPINA10 gene, fibrinogen gamma gene; PROC gene, and KNG1 gene. Candidate SNPs are Tagging SNPs for the gene. The selection method is based on the genome-wide SNP genotype data of Chinese people in the Hapmap database (http://www.hapmap.org), and Haploview software is used for LD analysis and Tagging SNP selection. Allele frequency ≥0.10, *r*2 ≥ 0.8 standard selection. Finally, 21 gene loci are selected for detection: FII gene rs3136447, rs5896, rs1799963 locus; FV gene rs6427199, rs2227245, rs6025, rs118203905, rs118203906 locus; FXI gene rs2289252, rs2036914 locus 20; F XIII gene rs5985; MTHFR gene rs1801133; ABO non-O type rs8176719, rs514659; SERPINC1 gene rs121909548; SERPINA10 gene rs2232698; fibrinogen gamma gene rs2066865; PROC gene rs1799810; KNG1 gene rs710446 site. The selected Tagging SNPs are genotyped by Sequenom MassARRAY detection technology.

RETRACTED

### 3.3. Experiment Group Design

#### 3.3.1. Experiment Grouping of Risk Factors for Hereditary Thrombophilia or/and VTE-Related Risk Factors

Case group selection follows the principles below: PC, PS, AT-III, and APCR indexes are lower than the normal range, and Hcy is higher than the normal value range. Any one of them is the hereditary thrombophilia population, including all deep vein thrombosis diagnosed by B-ultrasound from patients.

Control group selection follows the principles below: PC, PS, AT-III, and APCR indexes are in the normal range, Hcy is higher than the normal range, and there is not any of the exclusion conditions in the survey subjects, and they are included in the control group.

#### 3.3.2. Analysis of the Influence of Environmental Factors on Hereditary Thrombophilia

Case group selection follows the principles below: PC, PS, AT-III, and APCR indexes below the normal value range and Hcy above the normal value range, without any of the exclusion conditions, are included in the case group.

Control group selection follows the principles below: PC, PS, AT-III, and APCR indexes are in the normal value range, Hcy is in the normal value range, there is not any of the exclusion conditions in the survey subjects, and they are included in the control group.

### 3.4. SNP Mass Spectrometry Method Flow

#### 3.4.1. Reagent Preparation

Remove 10x PCR buffer, MgCl_2_, dNTP, and primers from −20°C and dissolve at room temperature. Store HotstarTaq at −20°C and take them out for use.

#### 3.4.2. PCR Reaction

The specific steps of PCR reaction are as follows:

1. Prepare a 384-well reaction table based on the extracted samples, and indicate the number of the DNA sample corresponding to each well and the primers used.
2. Add 1 *µ*L of DNA template to each well of the 384-well plate according to the table, paste the membrane, and centrifuge at 2000 rpm/10 seconds before use.
3. Prepare the PCR reaction solution as follows (take 384 samples as an example), and Table 1 shows the PCR reaction solution preparation.
4. Take a row of 12 tubes, add 133 *µ*L of the prepared PCR reaction solution to each well, and centrifuge briefly for later use.
5. Use a 10 ul spray gun to take 4 ul of PCR reaction solution from 12 tubes and add it to a 384-well plate containing 1 ul of DNA, so that the final volume of each well is 5 ul. Be careful that the pipette tip does not touch the DNA sample in the 384-well plate; if it does, the pipette tip needs to be replaced.
6. Briefly centrifuge the 384-well plate containing 5 ul of the reaction solution, put it into the PCR machine, and run the reaction program.
7. After the PCR reaction program is over, centrifuge the 384-well plate briefly for later use, and store it at 4°C.

RETRACTED

#### 3.4.3. SAP Processing

The specific steps of SAP processing are as follows:

1. Prepare the SAP reaction solution in the following order (take 384 samples as an example).  Table 2 shows SAP reaction solution preparation parameters.
2. Take a row of 12-tube tubes, divide the SAP reaction solution into 66 *µ*L per well, centrifuge briefly, and then dispense it into a 384-well PCR reaction plate with a 10 ul pipette, add 2 *µ*L to each well, seal with membrane, and centrifuge.
3. Put the 384-well plate into which the SAP reaction solution has been added into the PCR machine, and run the reaction program.
4. When the reaction is over, take out the 384-well plate and centrifuge briefly for later use.

#### 3.4.4. Extension Reaction

The specific steps of extension reaction are as follows:

1. Prepare iPlex reaction reagents.  Table 3 shows iPlex reaction reagent preparation.
2. Take a row of 12 tubes, aliquot the iPlex reaction solution in 66 *µ*L per well, centrifuge briefly, and then dispense it into a 384-well PCR reaction plate with a 10 ul pipette, add 2 *µ*L to each well, seal with membrane, and centrifuge.
3. Put the 384-well plate with the iPlex reaction solution into the PCR machine, and run the reaction program.
4. When the reaction is over, take out the 384-well plate and centrifuge briefly for later use.

#### 3.4.5. Product Purification

The specific steps of product purification are as follows:

1. Take 6 mg of resin on a 384-well resin scraper, cover it evenly, scrape off the excess resin, and leave it for 20 minutes.
2. Centrifuge the finished 384-well plate at 1000 rpm for 1 min, add 25 *µ*L of deionized water to each well, invert on the resin plate (be careful to fix it, it cannot be displaced), then invert the resin plate to the 384-well plate. The resin is dropped into a 384-well plate, and the membrane is sealed.
3. Take the long axis of the 384-well plate as the axis, invert the 384-well plate for 20 minutes, centrifuge at 3500 rpm for 5 minutes, and then set aside.

RETRACTED

#### 3.4.6. Detections

The detections include Nanodispenser SpectroCHIP chip spotting, MassARRAY Analyzer Compac mass spectrometry detection, and TYPER software which analyzes the experimental results and obtains typing data. During the phase of Nanodispenser SpectroCHIP chip spotting, the assay samples are transferred from the 384-well reaction plate to the MassARRAY SpectroCHIP chip covered with matrix. After the sample is transferred to the SpectroCHIP chip, it can be put into the mass spectrometer for detection. It only takes 3–5 seconds for each detection point, and the analysis is fully automatic.

## 4. Experimental Results and Analysis

### 4.1. Prevalence of Venous Thromboembolism among Kazak Pregnant Women

According to the inclusion and exclusion criteria of this paper, among the 976 Kazak pregnant and lying-in women volunteers, the average age is (27.22 ± 8.4), and the total prevalence of genetically related venous thromboembolism in the 976 Kazak pregnant and lying-in women is 330; the prevalence rate is 33.8.0% (basically consistent with the 2011–2013 National Natural Research data)—the prevalence of venous thromboembolism in Xinjiang Kazak pregnant and lying-in women, AT-III deficiency, PC deficiency, PS deficiency, APCR, and the prevalence of high homocysteine. Statistical analysis results are shown in Table 4.

### 4.2. The Results of Mass Spectrometry SNP Detection in Xinjiang Kazak Pregnant and Lying-In Women with Venous Thromboembolism

The assay samples are transferred from the 384-well reaction plate to the MassARRAY SpectroCHIP chip covered with matrix. Use MassARRAY Analyzer Compac mass spectrometry detection, and then transfer the sample to the SpectroCHIP chip, and then put it into the mass spectrometer for detection. It only takes 3–5 seconds for each detection point, and the automatic analysis is performed. The statistics of the detection results of each gene location are shown in Table 5.

The expression results of its alleles in the experimental group and the control group are counted, and the results are shown in Table 6. From the above experimental results, the whole SNP measurement results have obvious differences. Based on the results, we can further analyze the correlation between the polymorphisms in the promoter region and coding region of the TAFI gene of TAFI gene in Xinjiang Kazak pregnant and lying-in women and thrombosis or/and VTE. Statistical analysis is performed.

RETRACTED

### 4.3. Association of TAFI Gene Promoter and Coding Region Polymorphisms with Thrombophilia or/and VTE

In the correlation analysis between FII gene polymorphism and Kazak gene inheritance in pregnancy period venous thromboembolism, the gene frequency and allele frequency distribution are compared. The distribution of genotype frequency and allele frequency conformed to Hardy–Weinberg equilibrium (*P* > 0.05), indicating that the gene frequency reached a genetic balance and is representative of the population. Compared with the normal control group, there is a statistically significant difference in the allele frequency of rs3136447 in the hereditary thrombophilia patient group (*P* value = 0.0483), and there is also a statistically significant difference in the allele frequency of the rs5896 locus (*P* value = 0.0302). In addition, there is no significant difference in the distribution of the genotype and allele frequencies of the other loci among the groups, and the results are shown in Table 7. The data outside the brackets are examples, the data in the brackets are the composition ratio (%), the *P* value is calculated using *χ*^2^ and Fisher's exact test, and some variables are missing.

### 4.4. Analysis of the Interaction between Venous Thromboembolism and Environmental Factors in Kazak Pregnant and Lying-In Women

According to the experimental method in this paper, the indexes of PC, PS, AT-III, and APCR are lower than the normal value range, and Hcy is higher than the normal value range. Any one of them is the hereditary thrombophilia population, including all those diagnosed by B-ultrasound. Patients with deep vein thrombosis (experimental group) and those whose PC, PS, AT-III, and APCR indexes are in the normal range and Hcy higher than the normal range (control group) are surveyed by questionnaire. Drinking water, fresh meat, fresh vegetables, fresh fruit, salted meat, body mass index (BMI): weight/height 2 (kg/m^2^), and other patient's own and external environmental factors are investigated. For analysis, as shown in Table 8, the scoring statistics are carried out.

There are significant differences in the prevalence of some populations among the characteristic populations under different environmental factors, and the results are shown in Table 9.

At the same time, logistic regression analysis is carried out, and the results are shown in Table 10. OR value < 1 indicates that the factor is a protective factor. Otherwise, OR value > 1 indicates that the factor is a risk factor.

RETRACTED

## 5. Conclusions

To reveal the correlation between the prevalence of venous thromboembolism in Kazak pregnant and lying-in women in Xinjiang, the logistic regression additive model method is used to explore the interaction between the variation of two polymorphic loci and environmental factors. Through the measurement and analysis of anticoagulation indexes in 976 Kazak pregnant and lying-in women, it is found that the prevalence rate of venous thromboembolism in the pregnancy period related to genetic inheritance of Xinjiang Kazak pregnant and lying-in women is 33.8%, among which AT-III deficiency, the prevalence of PC deficiency, PS deficiency, APCR, and Hcy are 17.5%, 16.7%, 22.0%, 23.7%, and 26.8%, respectively. And from the two aspects of the interaction between the TAFI gene promoter region and coding region polymorphism, the correlation of venous thromboembolism in pregnancy period, and the interaction of environmental factors, the following conclusions can be drawn. The experimental result demonstrates that the GG type at the rs6427199 site of FV and the TT type at the rs2227245 site may be associated with antithrombin III deficiency in the Kazak population in Xinjiang, China.

## Figures and Tables

**Table 1:** PCR reaction solution preparation.

Reagent name	1 rxn (*µ*L)	384 rxn (*µ*L)
H_2_O	0.95	380
PCR buffer (10x, 含15 mM MgCl_2_)	0.625	250
MgCl_2_ (25 mM)	0.325	130
dNTP (2.5 mM each)	1	400
Primer solution	1	400
HotstarTaq (5 U/*µ*L)	0.1	40
Final volume	4	1600

**Table 2:** SAP reaction solution preparation parameters.

Reagent name	1 rxn (*µ*L)	384 rxn (*µ*L)
H_2_O	1.53	612
SAP buffer (10x)	0.17	68
SAP enzyme (1 U/*µ*L)	0.3	120
Final volume	2	800

**Table 3:** iPlex reaction reagent preparation.

Reagent name	1 rxn (*µ*L)	384 rxn (*µ*L)
H_2_O	0.755	302
iPlex buffer (10x)	0.2	80
iPlex termination mix	0.2	80
Primer solution	0.804	321.6
iPlex enzyme	0.041	16.4
Final volume	2	800

**Table 4:** Mean values and prevalence of AT-III, PC, PS, APCR, and Hcy among Kazak pregnant and lying-in women in Xinjiang.

Project	Case group 330	Control group 646	Total	Case	Prevalence
AT-III	68.34% ± 13.62%	88.34% ± 18.62%	78.24% ± 17.62%	171	17.5
PC	63.90％ ± 11.31%	92.90％ ± 28.31%	82.60％ ± 26.31%	163	16.7
PS	45.02％ ± 12.22%	65.02％ ± 20.22%	60.12％ ± 23.02%	215	22.0
APCR	>300 s	120–300 s		231	23.7
Hcy	15.37 ± 0.21%	9.23 ± 0.21%	11.23 ± 0.21%	265	26.8
Genetically related venous thromboembolism in Imchen period				330	33.8

**Table 5:** The detection results of different gene loci of mass spectrometry SNP in Kazak pregnant and lying-in women with venous thromboembolism in Xinjiang.

Gene locus	Frequency	Percentage	Effective percentage	Cumulative percentage
	2	0.0	0.0	0.0
A	382	7.3	7.3	7.3
AG	101	1.9	1.9	9.2
C	1630	31.1	31.1	40.3
CA	45	0.9	0.9	41.2
CT	249	4.7	4.7	45.9
DEL	97	1.8	1.8	47.8
DEL.C	128	2.4	2.4	50.2
G	890	17.0	17.0	67.2
GA	430	8.2	8.2	75.4
T	626	11.9	11.9	87.3
TA	109	2.1	2.1	89.4
TC	555	10.6	10.6	100.0
Total	5244	100.0	100.0	

RETRACTED

**Table 6:** The difference statistics of allele expression results between the experimental group and the control group.

Grouping		Statistic	Bootstrap^a^			
			Deviation	Standard error	95% confidence interval	
					Lower limit	Upper limit
Test group	Mean	1.8578	−0.0016	0.0411	1.7774	1.9381
	*N*	90		7	77	104
	Standard deviation	0.37837	−0.00362	0.02265	0.33136	0.41911
	Variance	0.143	−0.002	0.017	0.11	0.176

Control group	Mean	0.8075	0.0007	0.0381	0.7377	0.8856
	*N*	330	2	127	176	330
	Standard deviation	0.36662	−0.00213	0.02546	0.31388	0.41973
	Variance	0.134	−0.001	0.019	0.099	0.176

Total	Mean	1.3326	−0.0005	0.0483	1.2354	1.4274
	*N*	646	0	0	646	646
	Standard deviation	0.64448	−0.00322	0.02332	0.59306	0.68844
	Variance	0.415	−0.004	0.03	0.352	0.474

**Table 7:** Comparison of genotype and allele frequency of each locus in control group and case group.

Locus	Case group (330)	Control group (646)	*χ * ^2^	*P* value
rs3136447				
CC	55	92		
CT	142	283		
TT	133	271		
C	201	477	3.95	0.01 < *P* < 0.05
T	459	815		

rs5896				
CC	122	328		
CT	140	279		
TT	68	39		
C	386	897	11.72	*P* < 0.01
T	274	395		

**Table 8:** Questionnaire scoring criteria.

Project	Assign points
Age	
Less than 35 years old	1
35+	2
High blood pressure	The diagnosis of hypertension in hospitals above the county level is the standard

Drinking water	
Tap water	1
Hand press well	2
River, river water, mountain spring water	3

Fresh meat intake	
Not eating or less than 1 kg per month	1
1 kg to 2 kg per month	2
2 kg and above per month	3

Intake of fresh vegetables	
More than 2 kg per month	1
1 kg to 2 kg per month	2
Not eating or less than 1 kg per month	3

Fresh fruit intake	
More than 2 kg per month	1
1 kg to 2 kg per month	2
Not eating or less than 1 kg per month	3

Salted meat intake	
Not eating or less than 1 kg per month	1
1 kg to 2 kg per month	2
More than 2 kg per month	3

**Table 9:** Statistical analysis results of the correlation between venous thromboembolism and environmental factors in Kazak pregnant and lying-in women.

Characteristic factor	Characteristic number	Number of sick people	Prevalence %	Chi-square value	*P* value
Age				19.59	˂0.01
35−	844	263	31.2		
35+	132	67	50.7		

Hypertension				0.50	˃0.05
Have	235	75	31.9		
None	741	255	34.4		

Drinking water				4.55	˃0.05
Tap water	589	187	31.7		
Hand press well	267	93	34.8		
River, river water, mountain spring water	120	50	41.7		

Fresh meat intake				13.61	˂0.01
Not eating or less than 1 kg per month	73	22	30.1		
1 kg to 2 kg per month	230	56	24.3		
2 kg and above per month	673	252	37.4		

Intake of fresh vegetables				66.60	˂0.01
2 kg and above per month	360	89	24.7		
1 kg to 2 kg per month	336	92	27.3		
Not eating or less than 1 kg per month	280	149	53.2		

Fresh fruit intake				4.0466	˃0.05
2 kg and above per month	301	112	37.2		
1 kg to 2 kg per month	396	136	34.3		
Not eating or less than 1 kg per month	279	82	29.3		

Salted meat intake				5.26	˃0.05
Not eating or less than 1 kg per month	663	223	33.6		
1 kg to 2 kg per month	180	71	39.4		
2 kg and above per month	133	36	27.0		

RETRACTED

**Table 10:** Multivariate logistic regression analysis of genetically related Kazak pregnant and lying-in women on the prevalence of venous thromboembolism in the Imchen period.

Factor	*β*	S	*P* value	OR (95％ CI)
Age (1, 2)	0.597	0.230	˂0.01	1.818 (1.157–2.854)
Reduced intake of fresh vegetables (1, 2, 3)	0.215	0.163	˃0.05	1.240 (1.052–1.402)
Increased intake of fresh meat (1, 2, 3)	2.002	0.230	˂0.01	7.403 (4.716–11.621)

## Data Availability

The simulation experiment data used to support the findings of this study are available from the corresponding author upon request.
